The article "Morphological Characteristics of Young and Old Murine Hematopoietic Stem Cell Niches, as Modeled In Vitro" was published in 2023. Journal: Scanning.

# Morphological Characteristics of Young and Old Murine Hematopoietic Stem Cell Niches, as Modeled *In Vitro*

**DOI:** 10.1155/2023/5541050

**Published:** 2023-04-15

**Authors:** Mojca Justin, Ema Rogač Randl, Veno Kononenko, Matej Hočevar, Damjana Drobne, Primož Rožman

**Affiliations:** ^1^Blood Transfusion Centre of Slovenia, Ljubljana 1000, Slovenia; ^2^Department of Biology, Biotechnical Faculty, University of Ljubljana, Ljubljana 1000, Slovenia; ^3^Institute of Metals and Technology, Ljubljana 1000, Slovenia

## Abstract

The hematopoietic stem cell (HSC) niche undergoes detrimental changes with age. The molecular differences between young and old niches are well studied and understood; however, young and old niches have not yet been extensively characterized in terms of morphology. In the present work, a 2D stromal model of young and old HSC niches isolated from bone marrow was investigated using light and scanning electron microscopy (SEM) to characterize cell density after one, two, or three weeks of culturing, cell shape, and cell surface morphological features. Our work is aimed at identifying morphological differences between young and old niche cells that could be used to discriminate between their respective murine HSC niches. The results show several age-specific morphological characteristics. The old niches differ from the young ones in terms of lower cell proliferating capacity, increased cell size with a flattened appearance, increased number of adipocytes, and the presence of tunneling nanotubes. In addition, proliferating cell clusters are present in the young niches but not in the old niches. Together, these characteristics could be used as a relatively simple and reliable tool to discriminate between young and old murine HSC niches and as a complementary approach to imaging with specific cellular markers.

## 1. Introduction

The stem cell niche is a specialized microenvironment with a specific anatomy and function that regulates and maintains particular kinds of stem cells [1]. The most studied stem cells are hematopoietic stem cells (HSCs), which reside in the bone marrow niche. It is widely accepted that HSCs give rise to a complete set of immune and blood progenitors and that signals from the niche environment regulate HSC fate [2]. The HSC niche is a complex physiological environment composed of three main constituents: (a) HSCs and their differentiated myeloid and lymphoid progenitors; (b) a variety of stromal cells, including osteoblasts, osteoclasts, adipocytes, endothelial cells, mesenchymal stromal cells (MSCs), endothelial and perivascular cells, and macrophages; and (c) extracellular matrix, containing various molecules such as fibronectin, laminin, collagen, and a plethora of other components, such as chemoactive compounds, signaling molecules of the nervous system, hormones, cytokines, growth factors, and other molecules. Each of them plays a role in regulating self-renewal, proliferation, HSC differentiation, and HSC population maintenance [3, 4]. Due to the vital role of neuroendocrine and immune factors, some authors use the expression “HSC synapse” when speaking of the HSC niche (Figure 1). Signals from the stroma and other niche constituent cells can reach HSCs directly via cell-cell contacts through gap junctions or adhesion receptors, as well as via paracrine factors in the extracellular matrix [5].

It is known that the hematopoietic system undergoes substantial detrimental changes with age due to a combination of intrinsic and extrinsic factors which manifest as morphological changes to the HSC niche [6]. Briefly, cell-intrinsic alterations and underlying molecular mechanisms that lead to age-related defects of HSCs include (a) exhaustion of the stem cell pool, resulting in an inability to regenerate tissues, (b) telomere shortening with consequent cell senescence, (c) changes to microRNAs responsible for regulating the posttranscriptional expression of target genes, (d) DNA damage and mutations together with epigenetic changes, which can lead to the (e) loss of cell polarity and proteostasis, along with (f) a decline in mitochondrial function, accompanied by a decline in biogenesis. Lastly, (g) changes in metabolism and nutrient sensing occur, where signaling pathways involved in anabolic processes accelerate the aging of HSCs. Intrinsic cellular alterations have been extensively reviewed in several studies [7–10].

All of the intrinsic detrimental changes in aged HSCs listed above result in a decreased ability for self-renewal and myeloid-biased differentiation at the expense of lymphopoiesis [11]. Consequently, an increased number of myeloid leukemia cases and a decreased adaptive immune system are observed in the elderly [12, 13].

Apart from intrinsic changes, extrinsic factors such as cytokines, growth factors, hormones, and extracellular matrix in the niche also play a role in the HSC aging process. However, knowledge regarding the specific role of these factors in aging is far less extensive [6].

The molecular mechanisms that cause detrimental effects in aging HSCs are similarly active in other constituents of the niche, resulting in decreased osteogenesis and increased adipogenesis [3], nerve degeneration [14], and impaired endothelial cell function, with consequent loss of vascular integrity and higher microvascular permeability [11]. The most apparent change in the aged stroma is increased adipogenesis, as adipocytes eventually take up the majority of bone marrow (BM) volume [3]. This change is most likely a consequence of intrinsic changes in old MSCs (e.g., changes to the genome, transcriptome, and proteome), reduced concentrations of certain hormones (sex and pituitary hormones), and other factors in the blood plasma [15, 16].

Similarly, extracellular matrix components secreted mainly by niche stromal cells undergo specific aging-related changes. For example, the matrix becomes stiffer due to decreased collagen formation and secretion and a higher mineral phosphate content [17]. Age-related alterations in the HSC niche also affect soluble mediators, such as osteopontin, CXC-chemokine ligand 12, and CC-chemokine ligand 5 [10, 18, 19].

One morphological feature expected to enable the discrimination of cells between young and old niches is tubular membrane structures called tunneling nanotubes (TNTs). TNTs are thin, membranous cellular protrusions filled with cytoskeletal filaments (F-actin) that extend from the plasma membrane and enable intercellular connections over long distances [20]. TNT diameters range from 50 to 200 nm and can reach lengths over 100 *μ*m, while their morphology and composition can vary between and within cell systems [20]. They can transfer cytoplasmic material and organelles between cells [21, 22]. They also act as intercellular bridges that play a unique role in tissue repair and inflammation response, embryonic development, collective cell migration, injured cell recovery, cancer treatment resistance, and pathogen propagation [23]. Despite the ubiquitous observation of TNTs in cell cultures, only a few studies have described this phenomenon *in vivo* or in situ [24]. The significance of TNT biogenesis is unknown, but cells may need these unique structures in specific physiological circumstances to establish a means of intercellular communication not accomplished by other types of intercellular connections.

Understanding the underlying differences between young and aged hematopoietic stem cell niches is crucial for understanding the contributing factors that play a role in facilitating the aging process of HSCs. While there is a significant insight into the different molecular mechanisms that exist in young and aged stem cell niches, extensive morphological analysis of these differences has not been done before.

In this work, we isolated BM cells and cultured them as a 2D model of the niche. Light microscopy (LM) and scanning electron microscopy (SEM) were used to characterize cell shape, proportions of cells with different shapes, and their specific morphological features in 2D models of young and old murine HSC niches. We have focused on the stromal components of the bone marrow niche, composed of matrix components and stromal cells that are nonhematopoietic in nature and can be differentiated into multiple cell lineages. The aim of our work was to identify the morphological characteristics which could be used as a tool for discriminating between young and old murine HSC niches.

## 2. Materials and Methods

### 2.1. Animals

Young (11–12 weeks) and old (65-87 weeks) C57BL/6j mice were kept under controlled, pathogen-free conditions at the Medical Experimental Centre (MEC) in the Faculty of Medicine at the University of Ljubljana. The mice were housed in a 12 h light/dark cycle, with *ad libitum* access to food and water. In total, seven young and eight old mice were used, and each animal was taken as one biological repetition. The use of animals was approved by the Ethical Committee for Laboratory Animals of the Republic of Slovenia (No. U34401-27/2013/13), which is part of the Administration of the Republic of Slovenia for Food Safety, Veterinary, and Plant Protection.

### 2.2. Isolation and Cultivation of Bone Marrow (BM) Cells as a Hematopoietic Stem Cell (HSC) Niche Model

The mice were sacrificed using CO_2_ asphyxiation followed by cervical dislocation. For BM cell isolation, we used the bone crush method. We initially tried an isolation protocol with enzymes (collagenase); however, the isolated cells were of lower viability (66%) in comparison with the bone crush method, where enzymes were not used (95.1%) [25]. Furthermore, cell suspensions isolated with collagenase showed an increased concentration of debris and changes in cell morphology. For these reasons, we decided to use the bone crush method for isolating the BM cells, which we previously optimized [26]. In short, once the mice were euthanized, the bones (tibia, femur, humerus, ilia, and vertebrae) were collected, thoroughly cleaned, and crushed with a mortar and pestle together with a cold isolation medium (RPMI-1640 medium, Gibco, Grand Island, NY; 25 mM HEPES, Gibco; 1 mM EDTA, Gibco; 1x PenStrep, Gibco). Cell suspensions were then filtrated through a 40 *μ*m nylon cell strainer (Thermo Fisher Scientific) and centrifuged to remove remaining bone fragments. Once isolated, the cells were cultured according to the procedure used in the *Murine Long-Term Culture Initiating Cell (LTC-IC) Assay*. Once the pellet was obtained, the cells were resuspended in a commercial long-term culture medium (LTCM; MyeloCult™ M5300 with 10^−6^ M hydrocortisone), optimized to grow adipocytes, fibroblasts, and endothelial cells, and seeded into a 12-well plate at a density of 1 − 1.5 × 10^6^ cells per cm^2^ [27]. Before plating, sterile cover glasses were placed into each individual well to serve as a surface for cells to attach for further SEM analysis. The cells were then cultured for 1–3 weeks in an incubator at 33°C in 5% CO_2,_ and every week, half of the LTCM was replaced with fresh medium in every well. The process of artificial HSC niche preparation is presented in Figure 2.

### 2.3. Light Microscopy

Cell cultures from each animal were analyzed every week with a phase-contrast light microscope (Nikon) and computer program for image capturing (NIS-Elements) by placing the 12-well plates under the microscope. This was done to ensure that the cells developed properly and formed adherent stromal layers. Moreover, the cultures were checked to ensure the absence of contamination, which is seen as small unadhered particles in the medium.

### 2.4. Cell Density Assessment

After one, two, and three weeks of culturing, cell density in the young and old niches was determined from SEM micrographs using the ImageJ software (National Institutes of Health, Bethesda, MD, USA). For each week, at least two biological repetitions (samples from two mice) were used, where the number of cells was determined on an area of at least 2.5 mm^2^.

### 2.5. Sample Preparation and SEM Analysis

Cover glasses with attached cells were removed from culture plates every week for three weeks (*n* = 3). The cells were immediately rinsed in a fixative, as described by Hočevar et al. [28]. First, the samples were fixed with the Karnovsky fixative composed of 2.5% glutaraldehyde (SPI Supplies, West Chester, PA, USA) and 0.4% paraformaldehyde (Merck KGaA, Darmstadt, Germany) in 1 M Na-phosphate buffer (NaH_2_PO_4_·2H_2_O and Na_2_HPO_4_·2H_2_O; pH 7.3; Merck KGaA, Darmstadt, Germany) for 24 hours in a refrigerator. After fixation, the fixative was removed, and samples were washed with 1 M Na-phosphate buffer, followed by 60 min postfixation with 1% osmium tetroxide (OsO_4_) (SPI Supplies, West Chester, PA, USA). Samples were dehydrated in an ethanol series starting with 30% ethanol (EtOH; Merck KGaA, Darmstadt, Germany; 10 min), 50% EtOH (at least 10 min), 70% EtOH (at least 10 min), 80% EtOH (at least 10 min), 90% EtOH (at least 10 min), and absolute EtOH (at least 10 min). Further dehydration steps were performed with a mixture of hexamethyldisilazane (HMDS; SPI Supplies, West Chester, PA, USA) and absolute EtOH (1 : 2, *v*/*v*, 10 min; 1 : 1, *v*/*v*, at least 10 min) and with absolute HMDS, which was finally left to evaporate for 24 h. Samples were sputter-coated with gold/palladium using a precision etching coating system (682 PECS, Gatan, Pleasanton, USA) and examined with a field emission scanning electron microscope (SEM, JEOL JSM-6500F). SEM was used to visualize the attachment pattern, number, density, and morphology of adhered cells on the cover glass.

### 2.6. Statistical Analysis

All numerical data are expressed as arithmetic means + standard deviations (SD) and were statistically analyzed using the GraphPad Prism software (GraphPad Software, San Diego, CA). For comparison of cell density and distribution of different morphological cell types in the young and old murine HSC niches, ANOVA was used with Bonferroni's post hoc test. For comparison of the size of the flattened cells in the young and old HSC niches, the nonparametric Mann–Whitney *U* test was used. The difference between groups was considered statistically significant if the *p* value was less than 0.05.

## 3. Results

### 3.1. Different Cell Types of HSC Niche

Before SEM analysis, cell cultures were monitored using a light microscope to validate the formation of an artificial HSC niche. The main cell types of the HSC niche were identified based on previous reports, which include adipocytes (containing lipid droplets, Figure 3(a)), fibroblast-like cells (flattened and elongated, Figure 3(b)), and endothelial cells (growing in a line, Figure 3(c)). Therefore, light microscopy results confirmed the formation of the HSC niche *in vitro* after four weeks of culturing.

### 3.2. Cell Density

Results showed a higher density of BM stromal cells (adipocytes, fibroblast-like cells, and endothelial cells) in young niches already after one week of culturing in comparison to the old niches. However, the difference was not statistically significant. After two and three weeks of culturing, the difference in cell density became statistically significant, indicating a higher proliferating capacity of young BM cells in comparison with the old cells (Figures 4 and 5). In addition, emerging proliferating cell clusters in young niches were observed after one week of culturing (Figure 6).

### 3.3. Differences in Cellular Morphological Characteristics between Young and Old HSC Niches

Using SEM, we identified four predominant, morphologically distinct cell types in both HSC niches. These consist of flattened cells, round cells, adipocytes filled with lipid droplets (observed as round intracellular vesicles), and elongated cells with protrusions (Figure 7). In both young and old HSC niches, flattened cells were predominant. In the young HSC niches, the proportion of flattened cells was more than 50%, while in the old HSC niches, the portion of flattened cells was around 40%. The round cells made up about 20% of the cells in the young HSC niches and slightly more, about 25%, in the old HSC niches (Figure 8). The rest of the young and old HSC niche cells were elongated with protrusions of different sizes (explained in detail below). As expected, the most significant difference between the young and old HSC niches was in the proportion of adipocytes. We estimate that less than 5% of all cells were adipocytes in the young HSC niches, but for a more accurate estimate, large numbers of cells would need to be analyzed using immunostaining and flow cytometry, for example.

We also compared the average size of flattened cells in the young and old HSC niches. In the old HSC niches, the flat cells were significantly larger (Figure 9).

The most obvious characteristic of the old niche is the increased content of adipocytes that develop from MSCs. SEM micrographs reveal multiple adipocytes in the old niches (Figure 10). In the young niches, adipocytes are rarely seen (less than 5%).

Adipocytes show a high content of lipid droplets (Figure 11).

As expected, a morphological characteristic of cells in the old niches, as revealed by SEM analysis, is cells with tunneling nanotubes (TNTs). These are thin cytoplasmic extensions bridging two cells that are more than 100 *μ*m long. TNTs were only observed in the old HSC niche samples and were completely absent in the young HSC niche samples (Figure 12).

## 4. Discussion

Our study provides evidence that 2D models of young and old murine HSC niches have distinct morphological characteristics that can be used to discriminate between them on the basis of the shape and morphological attributes of stromal cells isolated from the respective young and old bone marrows. The young niches contained proliferating cell clusters, which were absent in the old niches. A lower total number of cells characterized the old niches after two and three weeks of culturing (highlighting the higher proliferative capacity of young niche cells), along with larger sizes of flattened cells, higher number of adipocytes, and the presence of cells with TNTs. It is worth noting that in this work, we isolated BM cells and cultured them as a 2D model of the niche, in which we only managed to grow some of the niche cells (endothelial cells, adipocytes, and fibroblast cells).

It was previously shown that old bone marrow (BM) cells have a lower proliferative capacity [5, 8], resulting in a lower cell density in the HSC niche. In our study, this was confirmed after two and three weeks of culturing. The higher proliferative capacity of the young niches was also demonstrated by the presence of proliferating cell clusters. After three weeks of culturing, maximum confluency was reached in the young niches, resulting in cell detachment and consequent death (seen as detached cell clusters in Figure 8). Light microscopy and SEM confirmed the presence of different cell types in the HSC niches. Our results demonstrated that the old niches had larger flattened cells, in line with literature reports. Various authors have provided evidence that aged mesenchymal stromal cells (MSC) in BM display an enlarged senescent-like morphology, delayed clonogenic potential, and reduced proliferative capacity compared to younger counterparts [25–27].

Our results also align with prior literature describing increased quantities of adipocytes in BM with aging. This phenomenon is known as “fatty degeneration,” where the adipocytes occupy almost the entire bone marrow space previously occupied by red hematopoietic marrow at a young age [29]. However, the role of adipocytes in BM is still largely unexplored [15, 16]. Age-associated adipocyte hypertrophy is associated with increased lipolysis, increased secretion of the leptin polypeptide and inflammatory cytokines, and decreased secretion of anti-inflammatory cytokines and adiponectin [30, 31]. It has been shown that an accumulation of adipocytes in aged BM inhibits both hematopoiesis and bone regeneration [17, 29]. In this work, we have shown that the presence of adipocytes, as observed by SEM, can be used to distinguish between young and old niches.

The final characteristic we observed that enables one to discriminate between young and old niches is the presence of tunneling nanotubes (TNTs) in some stromal cells of the aged HSC niches. It is assumed that there is a positive correlation between TNT development and cellular stress, in which cells may develop TNTs as a response to stress [20]. Moreover, TNT formation in association with immunity and inflammation has been reported in several studies in recent years [21, 32, 33]. TNTs have also been shown to present a way of communicating between senescent cells [34]. These authors report the contribution of TNTs toward the expression of senescence markers. Senescence is related to the cellular response to different physiological states, including stress, and is characterized by the permanent exit of the cell from the cell cycle.

## 5. Conclusions

We successfully identified morphological differences between young and old HSC niches. The differences with the highest discriminative power are

1. Increased proportion of adipocytes in the old niches (more than 25%)
2. Formation of TNTs by stromal cells in the old niches that were not observed in the young niches, and
3. Larger size of flattened cells in the old niches

Differences in the proportion of flattened and round-shaped cells between the young and old HSC niches were also observed but were not statistically significant. In addition, the old niches were characterized by a lower proliferative capacity, as expected.

The formation of TNTs by stromal cells in the old niches is a novel finding that has not yet been documented before and should be explored further. In addition, larger flattened cells are another morphological characteristic of old niches that indicates senescence. We conclude that the morphological features described in our study could be used as a tool to discriminate between young and old HSC niches. This is of particular interest when manipulations of stem cell niches are studied, such as seeding different combinations of cell types, adding bioactive molecules such as cytokines, or when anticipating adverse effects on a stem cell niche.

## Figures and Tables

**Figure 1:** Components of hematopoietic stem cell (HSC) niches (“HSC synapse”). Abbreviations: MSC: mesenchymal stem cells; Ecs: endothelial cells; HSCs: hematopoietic stem cells. Provided courtesy of P. Rožman.

**Figure 2:** Preparation of an artificial hematopoietic stem cell (HSC) niche. First, the bone crush method is used to isolate BM cells from young and old mice. The cells are then separately cultivated in a commercial MyeloCult medium for 1-3 weeks and regularly checked with light microscopy and SEM.

**Figure 3:** Light micrographs of representative cell types of a hematopoietic stem cell (HSC) niche investigated using a phase-contrast light microscope (200x) after four weeks of culturing. Adipocytes with lipid droplets, seen as round structures of different sizes, are indicated with a red arrow (a); fibroblast and mesenchymal stromal cells (MSCs) are characterized by a flattened and elongated shape (b); endothelial cells growing in lines are indicated with a blue arrow (c).

**Figure 4:** Cell density in young and old murine hematopoietic stem cell (HSC) niches after one, two, and three weeks of culturing. Data are presented as the mean number of cells per mm^2^ (+SD). An asterisk indicates a significant difference between young and old niches (^∗^ equals *p* < 0.05; ANOVA with Bonferroni's post hoc test).

**Figure 5:** SEM micrographs of young and old bone marrow (BM) niches after one week (a), two weeks (b), and three weeks of culturing (c). The proliferating cell clusters are seen in images (b) and (c) of the young niche (see detail in Figure 6).

**Figure 6:** Bone marrow cells from young mice after one week of culturing. The red square indicates a proliferating cluster. An example of a flattened cell is indicated with a yellow arrow, while an example of a flattened cell is indicated with a yellow asterisk.

**Figure 7:** SEM micrographs of different, morphologically distinct cell types in young and old hematopoietic stem cell (HSC) niches. (a–c) Flattened cells with a folded central area ((a, c) round; (b) oval) ((a, c) cells with a low number of short filopodia; (b) cell with a large number of filopodia) and differing cell surface roughness ((a, b) cells with rough membrane surfaces; (c) cell with smooth membrane surface). (d–f) Round-shaped cells with a large number of filopodia (d), extended lamellipodium (e), and visible cellular protrusions (f). (g) Adipocyte filled with numerous lipid droplets. (h) elongated cell. Scale bar = 10 *μ*m.

**Figure 8:** Relative distribution of different morphological cell types in young and old hematopoietic stem cell (HSC) niches. Data are presented as the mean percentage of all cells (+SD).

**Figure 9:** The average size of flattened cells in young and old hematopoietic stem cell (HSC) niches ± standard deviations (SD). Asterisk presents a significant difference between young and old niches (^∗^ equals *p* < 0.05; Mann–Whitney *U* test).

**Figure 10:** Adipocytes in an old niche are indicated with red arrows. A morphological characteristic of adipocytes is the presence of a large number of round intracellular vesicles (lipid droplets).

**Figure 11:** Multiple lipid droplets in adipocytes. Lipid droplets are intracellular organelles of varying sizes (from submicron dimensions to several microns) that can be seen as round-shaped structures beneath the cell surface in SEM imaging.

**Figure 12:** Tunneling nanotubes (TNTs) observed in an old hematopoietic stem cell (HSC) niche, indicated with a red arrow. TNTs were observed only in the old HSC niches.

## Data Availability

The data used to support the findings of this study are available from the corresponding author upon request.

## References

[1] Morrison S. J., Scadden D. T. (2014). The bone marrow niche for haematopoietic stem cells. *Nature*.

[2] Kumar S., Geiger H. (2017). HSC niche biology and HSC expansion _ex vivo_. *Trends in Molecular Medicine*.

[3] Latchney S. E., Calvi L. M. (2017). The aging hematopoietic stem cell niche: phenotypic and functional changes and mechanisms that contribute to hematopoietic aging. *Seminars in hematology*.

[4] Zhang C. C., Lodish H. F. (2008). Cytokines regulating hematopoietic stem cell function. *Current Opinion in Hematology*.

[5] Geiger H. (2012). Aging of the niche and the microenvironment and its role in stem cell aging. *Advances in Stem Cell Aging*.

[6] Woolthuis C. M., de Haan G., Huls G. (2011). Aging of hematopoietic stem cells: intrinsic changes or micro-environmental effects?. *Current Opinion in Immunology*.

[7] Rožman P. (2018). The potential of non-myeloablative heterochronous autologous hematopoietic stem cell transplantation for extending a healthy life span. *Geroscience*.

[8] Jazbec K., Jež M., Justin M., Rožman P. (2019). Molecular mechanisms of stem cell aging. *Slovenian Veterinary Research*.

[9] López-Otín C., Blasco M. A., Partridge L., Serrano M., Kroemer G. (2013). The hallmarks of aging. *Cell*.

[10] Guidi N., Sacma M., Ständker L. (2017). Osteopontin attenuates aging-associated phenotypes of hematopoietic stem cells. *The EMBO Journal*.

[11] Poulos M. G., Ramalingam P., Gutkin M. C. (2017). Endothelial transplantation rejuvenates aged hematopoietic stem cell function. *The Journal of Clinical Investigation*.

[12] Rossi D. J., Bryder D., Zahn J. M. (2005). Cell intrinsic alterations underlie hematopoietic stem cell aging. *Proceedings of the National Academy of Sciences*.

[13] Sudo K., Ema H., Morita Y., Nakauchi H. (2000). Age-associated characteristics of murine hematopoietic stem cells. *The Journal of Experimental Medicine*.

[14] Lazzari E., Butler J. M. (2018). The instructive role of the bone marrow niche in aging and leukemia. *Current stem cell reports*.

[15] Horowitz M. C., Berry R., Holtrup B. (2017). Bone marrow adipocytes. *Adipocytes*.

[16] Fazeli P. K., Horowitz M. C., MacDougald O. A. (2013). Marrow fat and bone—new perspectives. *The Journal of Clinical Endocrinology & Metabolism*.

[17] Ambrosi T. H., Scialdone A., Graja A. (2017). Adipocyte accumulation in the bone marrow during obesity and aging impairs stem cell-based hematopoietic and bone regeneration. *Cell Stem Cell*.

[18] Ergen A. V., Boles N. C., Goodell M. A. (2012). Rantes/Ccl5 influences hematopoietic stem cell subtypes and causes myeloid skewing. *Blood, The Journal of the American Society of Hematology*.

[19] Tuljapurkar S. R., McGuire T. R., Brusnahan S. K. (2011). Changes in human bone marrow fat content associated with changes in hematopoietic stem cell numbers and cytokine levels with aging. *Journal of Anatomy*.

[20] Zhang Y. (2011). Tunneling-nanotube: a new way of cell-cell communication. *Communicative & Integrative Biology*.

[21] Nawaz M., Fatima F. (2017). Extracellular vesicles, tunneling nanotubes, and cellular interplay: synergies and missing links. *Frontiers in Molecular Biosciences*.

[22] Ariazi J., Benowitz A., De Biasi V. (2017). Tunneling nanotubes and gap junctions–their role in long-range intercellular communication during development, health, and disease conditions. *Frontiers in Molecular Neuroscience*.

[23] Han X., Wang X. (2021). Opportunities and challenges in tunneling nanotubes research: how far from clinical application?. *International Journal of Molecular Sciences*.

[24] Shahar M., Szalat A., Rosen H. (2021). Pathogenic stress induces human monocyte to express an extracellular web of tunneling nanotubes. *Frontiers in Immunology*.

[25] Jazbec K. (2014). *Consecutive Bone Marrow Transplantation in Non-Irradiated Balb/c Mice*.

[26] Justin M., Jež M., Košir A., Miceska S., Rožman P., Jazbec K. (2021). Application of the 3R principles: vertebrae as an additional source of murine bone-marrow cells. *Laboratory Animals*.

[27] *Mouse Long-Term Culture-Initiating Cell (LTC-IC) Assay (2019). Manual [PDF file]*.

[28] Hočevar M., Batič B. Š., Godec M., Kononenko V., Drobne D., Gregorčič P. (2020). The interaction between the osteosarcoma cell and stainless steel surface, modified by high-fluence, nanosecond laser pulses. *Surface and Coatings Technology*.

[29] Naveiras O., Nardi V., Wenzel P. L., Hauschka P. V., Fahey F., Daley G. Q. (2009). Bone-marrow adipocytes as negative regulators of the haematopoietic microenvironment. *Nature*.

[30] Castro J. P., Grune T., Speckmann B. (2016). The two faces of reactive oxygen species (ROS) in adipocyte function and dysfunction. *Biological Chemistry*.

[31] Li Y., Meng Y., Xijie Y. (2019). The unique metabolic characteristics of bone marrow adipose tissue. *Frontiers in Endocrinology*.

[32] Campana S., De Pasquale C., Carrega P., Ferlazzo G., Bonaccorsi I. (2015). Cross-dressing: an alternative mechanism for antigen presentation. *Immunology Letters*.

[33] Önfelt B. Ö., Nedvetzki S., Yanagi K., Davis D. M. (2004). Cutting edge: membrane nanotubes connect immune cells. *The Journal of Immunology*.

[34] Whitehead J., Zhang J., Harvestine J. N., Kothambawala A., Liu G.-y., Kent Leach J. (2020). Tunneling nanotubes mediate the expression of senescence markers in mesenchymal stem/stromal cell spheroids. *Stem Cells*.

